# Computed Tomographic Image Processing and Reconstruction in the Diagnosis of Rare Osteochondroma

**DOI:** 10.1155/2021/2827556

**Published:** 2021-08-14

**Authors:** Ting Zhao, Hongyan Zhao

**Affiliations:** ^1^Department of Nursing, Shengjing Hospital of China Medical University, Shenyang, Liaoning 110004, China; ^2^Department of General Surgery, Shengjing Hospital of China Medical University, Shenyang, Liaoning 110004, China; ^3^Department of Orthopedics, Shengjing Hospital of China Medical University, Shenyang, Liaoning 110004, China

## Abstract

**Objective:**

We applied computed tomography (CT) to explore the imaging manifestations of rare parts of osteochondroma. Based on the medical images, deblurring using a convolutional neural network (CNN), and three-dimensional (3D) reconstruction of the images is performed in order to improve the image diagnosis.

**Methods:**

Twelve cases of osteochondroma in rare locations confirmed by surgical pathology or clinical long-term dynamic observation were retrospectively analyzed using medical imaging and image reconstruction. There are 7 males and 5 females, with an average age of 43 years. CT examinations were performed in all cases. Image deblurring via the GAN model is performed followed by the 3D reconstruction of the higher quality images is implemented. A retrospective study was performed on the imaging manifestations of the above cases; the imaging characteristics were summarized.

**Results:**

The imaging features are the following lesions, including 4 cases of the proximal radius, 4 cases of the scapula, 2 cases of the pelvis, and 2 cases of the proximal ribs. The cartilage caps, cortex, and sternum were typical structures of the bone surface of the studied cases. In the continuous imaging features, calcification was visible in some cases, and no significant enhancement was seen in enhanced scans; there was no obvious direction of lesion growth. The image processing techniques that we performed are useful in enhancing the quality of the medical diagnosis.

**Conclusions:**

Rare site osteochondroma has certain imaging features. In most cases, we can accurately diagnose rare site osteochondroma through these features via the image processing methods that are proposed in this paper.

## 1. Introduction

At present, the research in the field of image deblurring in the medical field mainly includes the medical image processing of data sets following the implementation of deblurring algorithms. In the field of medical deep learning, the status of image map data sets is self-evident, and the quality of the data set directly affects the quality of the experimental results. Compared with other image degradation and restoration problems, it is more difficult to obtain a data set for medical image deblurring, because it is difficult to capture a pair of clear images with exactly the same factors in a real lesion map, even if two consecutive images are taken. These two images will not correspond exactly due to changes in some factors, so it is almost impossible to obtain a pair of clear and blurred images with exactly the same content.

Osteochondroma is a common benign bone tumor in childhood. It is usually located on the cortex of one side of the metaphysis and grows to the surface of the bone. It is also called exoskeleton wart. Osteochondroma can be divided into single and multiple; the latter has a genetic predisposition and affects the development of epiphyseal or limb deformities, known as multiple hereditary osteochondroma disease, or continuation of the backbone. Lesions are located in the metaphysis, most commonly, the distal femur, the proximal tibia, and the proximal humerus. Clinically, osteochondroma has no pain or tenderness and produces corresponding symptoms when the nerve is compressed.

Osteochondroma is a common benign tumor in clinical work, accounting for 10-15% of all bone tumors and 20-50% of benign bone tumors. The ratio of male to female is 1.6 : 1 [1, 2], and the most common sites are the distal femur and the proximal tibia, followed by the proximal humerus, the distal radius, and the ends of the fibula, and can also occur in flat bones and other places [3]. This article focuses on the analysis of osteochondroma that occurs in flat bones, irregular bones, and proximal radiuses. Occurrence of osteochondroma in rare parts, due to its special location, generally does not attract the attention of clinicians; diagnostic experience is limited; in actual work, there are still diagnostic errors. This article summarizes the performance of 12 cases of osteochondroma in rare parts, and strives to improve the imaging diagnosis of osteochondroma in rare parts.

## 2. Materials and Methods

### 2.1. Convolutional Neural Network

Convolutional neural network is a classic deep learning network that promotes the rapid development of artificial intelligence. Convolutional neural network is composed of input layer, convolutional layer, activation function, pooling layer, and fully connected layer. Among them, the input layer is used to load the image with the input pixel size of *H* × *W* × *D* into the network; the convolution layer is used to extract image features; the input image and the convolution kernel should be multiplied by position elements and then summed, and finally, the convolution of the feature map after the product. In convolution operations, weight sharing is usually used to reduce the amount of calculation. Shared weights are different images or the same image sharing a convolution kernel. Using weight sharing can reduce the number of convolution kernels and speed up the training of the network. In order to better connect local information, convolution kernels generally use partial overlap sliding in the feature map to perform convolution operations. Overlap sliding means that there is an overlap between two adjacent convolution kernels. This sliding method makes the convolution calculation of the local receptive fields reduce the amount of calculation and at the same time ensures that there is a certain connection between the information extracted by the two local receptive fields. The neural network convolution operation is shown in Figure 1.

### 2.2. Patients Information

A retrospective study was performed to collect 12 cases of osteochondroma diagnosed in rare locations confirmed by surgical pathology or clinical follow-up observation. There were 7 males and 5 females, with an average age of 43 years. Ten patients were diagnosed with local palpitation, and two cases had lesions found during normal physical examination. All patients underwent CT examinations.

### 2.3. Indications for Surgery

Surgical treatment is performed for cases with obvious clinical symptoms, which include pain, limited joint movement, neurovascular compression, bursitis, or severely affected appearance. For patients with single-pedicled osteochondroma that occurs in the long tubular bones of the extremities, there are only regular follow-up observations if there are no clinical symptoms [4–6]. Consider surgical resection of osteochondroma with (1) clinical symptoms such as pain or discomfort; (2) fracture of the diseased pedicle; (3) local bursitis; (4) affecting joint activity; (5) compression of nerve blood vessels; (6) the lesions may increase in a short time or the symptoms may be aggravated; malignant changes may be suspected; (7) patients who affect the appearance strongly demand surgery. As for multiple osteochondroma, due to multiple lesions throughout the body, patients should be selected to perform surgery on the areas that affect them the most. Most of these areas seriously affect the appearance or joint activity and even cause joint deformities or they should be vigilant in the short term. Here, the malignant areas are seen to be existent.

Comparative analysis of the image characteristics includes the incidence of the case studied, the number of lesions, the shape of the cartilage cap, the density of the lesion, and the change in the density of the lesion after enhanced scanning, the condition of the adjacent bone cortex and bone structure, the direction of lesion growth, and the surrounding soft tissue. We summarize its imaging characteristics and improve the accuracy of diagnosis.

### 2.4. Surgical Resection Range

Longitudinal incision, separated to the surface of the mass, cut the bursa, cut the periosteum in a ring along 0.5~1 cm outside the base of the mass, cut the normal bone cortex of the host bone with a scalpel along this line, and then loosen along the bottom of the mass. Plasmas make sure to remove the fibrous membrane, cartilage cap, and bone warts outside the cartilage of the tumor together with the surrounding normal periosteum and cortical bone.

## 3. Results

### 3.1. Distribution of Lesions

In order to verify the effectiveness of the model, this paper explores the performance of the image motion blur removal model proposed in this paper from three aspects: visual effect, peak signal-to-noise ratio, and training time. The model in this article converges after being trained 200,000 times on the above training set, and the effect of the model is tested on the test set.

The effect of removing the blurred part of the image from the image in the data set is shown in Figure 2. On the left is the original blurred image in the data set, and on the right is the clear image generated after the model in this article. It can be seen from the experimental visual effects that the model proposed in this paper achieves a clear resolution of the visual effect of removing the blur of medical image images, and the calculation time of each step during training is increased by 0.04 seconds, and the test time is also reduced by 0.04 seconds.

This paper uses peak signal-to-noise ratio (PSNR) to measure the effect of image processing. The PSNR is an engineering term that represents the ratio of the maximum possible power of a signal to the destructive noise power that affects its representation accuracy. Since many signals have a very wide dynamic range, they are often expressed in logarithmic decibel units. The higher the peak signal-to-noise ratio, the higher the similarity between the restored image and the original image. This paper compares this metric with CNN-15, the deblurring method based on l0 norm, and our previous work SRN method. The experimental results are shown in Table 1.

The convergence of model training over time is shown in Figure 3.

Red represents the model in this paper, and blue represents the image blurring model based on the generative adversarial network in work. It can be seen that the model in this paper converges faster than the model in work.

There were 4 cases of proximal radius, 4 cases of scapula, 2 cases of pelvis, and 2 cases of proximal ribs (as shown in Table 2). There were 2 cases of the proximal radius (Figure 4), 4 cases of the scapula body, all located above the dorsal scapula (Figure 5), 2 cases of the pelvis (Figure 6), and 2 cases of the proximal rib (Figure 7). CT examinations were performed in all the studied cases to exclude possible osteochondroma lesions in other prevalent sites, and it was judged that the patients studied were single cases.

The middle part 4 of the proximal radius of the limb is shown, for example, in Figure 4 based on CT using medical images and 3D analysis based on the image reconstruction. There were 4 cases of scapula and 2 cases of pelvis in front of the scapula. The left mandibular angle is shown in Figure 5. The left mandibular coronoid process is shown in Figure 6. The proximal rib 2 is shown in Figure 7.

### 3.2. Cartilage Cap Morphology

The top of osteochondroma is covered with cartilage, called a cartilage cap, which varies in thickness. The thin ones are only linear translucent areas, which are not easy to see. The tumor surface of 7 patients who underwent the CT examination showed typical cartilage signals. Combined with CT and the 3D image reconstruction, 3 cases of spotted and strip-like calcifications were found inside the cartilage cap. The patients in this group are mainly sessile, the lesions are dish-shaped or hemispherical, and the apex is uneven, showing nodular and cauliflower-like changes. Lesion cartilage caps are small and well-defined, suggesting benign growth.

### 3.3. Changes in Lesions and Enhanced Scans

Of the 12 patients, 3 had punctate and strip-like calcifications inside the lesion, and the rest of the lesion had cartilage and changes in bone density or signal. There was no obvious abnormal enhancement in all lesions on the enhanced scan, indicating that the blood flow of the lesion was not abundant.

### 3.4. Near the Cortex and Bone Structure

All lesions showed signs of continuous connection with the adjacent normal bone (female bone) cortex. No obvious bone destruction and periosteal reaction were found in the adjacent bones.

### 3.5. Direction of Lesion Growth

Occurrence of osteochondroma in the proximal radius is a local bulge without obvious directionality. Osteochondroma of the scapula body showed a local bony hump in the posterior part of the scapula without obvious directionality. Pelvic chondroma grows outward. Two cases of rib osteochondroma occurred near the ribs and grew along the long axis of the ribs.

### 3.6. Surrounding Soft Tissue

In the studied case, the bone cortex was intact, there was no obvious swelling of the local soft tissue, and there was no abnormal density change inside. No abnormal enhancement was seen on the enhanced scan.

## 4. Discussion

### 4.1. The Etiology and Pathological Basis of Osteochondroma

Some studies conclude that osteochondroma is a real tumor, and some scholars suggest that it is caused by the lack of growth of the developmental epiphysis [7–9]. Virchow et al. proposed that a single osteochondroma is a tumor formed when the epiphyseal cartilage plate is separated and grows laterally outside the bone during development. Lithtenstein et al. believe that the periosteum develops abnormally, and the displaced cartilage nest continues to grow [10–13]. Osteochondroma is a three-layer typical structure: (1) the surface layer is collagen connective tissue with scarce blood vessels, which is connected with the surrounding periosteum and is closely attached to the underlying tissue; (2) the middle layer is gray-blue transparent cartilage, that is, “cartilage cap,” which is similar to normal cartilage and often calcified; (3) the base layer is the main body of the tumor, and the bone marrow containing yellow bone marrow is connected to the affected bone. In theory, osteochondroma can occur in any bone with cartilage internalized bone, an ossified form [12].

### 4.2. Advantages of General Radiography, CT, MRI, and Other Imaging Methods for Diagnosis

X-ray diagnosis is simple and easy. It is a basic examination method. It can initially determine the growth direction of osteochondroma lesions, internal calcification, and whether the cortex is connected. It has obvious advantages in the diagnosis of osteochondroma in the middle limbs. For areas with many overlapping areas, such as the pelvis, ribs, and scapula, further CT scans are needed to confirm. CT examination and three-dimensional reconstruction can clearly show the relationship between the tumor and the affected bone, showing that the lesion is continuous with the surrounding bone cortex, calcification of the cartilage cap of the lesion, and the condition of the surrounding soft tissue [13, 14]. Combined with the enhanced scan to judge the blood flow of the lesion, the diagnosis can be basically confirmed. It is the preferred method for the diagnosis of osteochondroma in rare sites; it is also helpful for the differential diagnosis of osteochondroma and periosteal chondrosarcoma.

MRI can also independently diagnose osteochondroma [15]. It can show the connection between the tumor and the affected bone from multiple angles. It can directly display the cartilage signal of the cartilage cap. MRI can also show changes in the bursa around the lesion. The basal periphery of the tumor on the MRI is a linear cortical bone connected to the normal female bone, with low signal on T1WI and T2WI; cancellous bone with fatty pulp in it, high signal on T1WI and moderate signal on T2WI; noncalcified cartilage. The appearance of the cap is leaf-shaped, containing uniform and consistent cartilage. T1WI is low signal, and T2WI is high signal. The calcified cartilage caps T1WI and T2WI are both banded or cauliflower-shaped low signal regions. The surface fibrous membrane is linear low signal [16, 17].

### 4.3. Differential Diagnosis

(1) Chondrosarcoma: It usually occurs in the long bones of the extremities. Most are thought to be related to embryonic tissue or ectopic, most of which are endogenous, exogeneous, or paracortical, tumors are lobulated and have fibrous envelopes, and the main component is hyaline cartilage. Homogeneous high-signal hyaline cartilage is separated by low-signal fibrous compartments and changes in leaf shape or uneven signal; the degree of malignancy is higher. In patients with multiple hereditary exostosis, the risk of malignant transformation into chondrosarcoma is greater. Chondrosarcoma is more likely if the thickness of the cartilage cap is greater than 2 cm [18].

(2) Malignant changes of osteochondroma: The main manifestations are as follows: (1) tumors grow rapidly; (2) the thickness of cartilage caps is greater than 1.0 cm or a large number of irregular calcifications; (3) the density of calcification of cartilage caps suddenly fades; translucent areas appear newly; soft tissue masses appear around the tumor, distant metastases from the tumor.

(3) Bone islands: It shows uniform density shadows in any part of the bone, mostly uniform high density shadows, that is, dense bone islands, and there are uniform low density shadow changes, such as osteoporotic bone islands. It is a common developmental mutation that is a benign change; however, it rarely rises from the growth of the cortical bone, and its uniform internal density is its characteristic.

### 4.4. Medical Image Processing Techniques Used in Medical Diagnosis

In recent years, with the popularization of imaging equipment and the large-scale use of digital images, the application value of image deblurring continues to increase, and many algorithms blindly improve the effect of removing image blur, but ignore the running time of the algorithm. In order to further improve the effectiveness and practicability of the algorithm, this paper combines a large amount of related work and proposes a model based on the generation of countermeasure network to remove image motion blur, which greatly improves the practicability of the model; on this basis, a further method based on convolutional neural network can be used to remove the image blurring.

In addition to the rare osteochondroma described in this paper, osteochondromas of the spine and clavicle have also been reported in the literature [19]. Among them, spinal osteochondroma is more common in spinal appendages, especially spinous processes.

In short, in addition to the common features of some common osteochondromas, the rare parts of osteochondroma combine with this group of cases and related literature [20].

## 5. Conclusion

This paper utilized 3D medical image reconstruction based on CT and summarizes the following characteristics: osteochondromas may appear in the scapula, proximal radius, and pelvis, rare parts such as ribs; the lesions are solitary; the broad bottom is connected to the female bone, the cortex continues from the female bone to the tumor, the outer edge is cortical bone connected to normal bone, and the inner is cancellous bone, which communicates with the mother's medullary cavity; the top is the structure of the cartilage cap. CT can show the presence of the cartilage cap; malignant changes are rare; there is no obvious direction of growth. Because there are few cases in this group, osteochondroma of all rare parts is not included, so the imaging study of rare parts of osteochondromas needs to be further studied and expanded. Furthermore, the 3D medical image diagnosis can be applied after superresolution image reconstruction is implemented so as to achieve a better quality image.

## Figures and Tables

**Figure 1:** Convolution neural network operation.

**Figure 2:** (a) changed to (b) is to remove the image blur state test effect diagram.

**Figure 3:** Convergence of model training over time.

**Figure 4:** Based on the 3D image reconstruction, the right radial bone is locally irregularly raised, the internal density is unevenly reduced, the CT lesion is continuous with the surrounding cortex, and the interior is cartilage density or signal.

**Figure 5:** Osteochondroma protruding from the left scapula posterolaterally after image deblurring.

**Figure 6:** Osteochondroma protruding from the right pelvis (sacrum) posterolaterally.

**Figure 7:** Osteochondroma of the right rib is continuously displayed around the outer cortex based on 3D reconstruction of the structure.

**Table 1:** Comparison of experimental results of peak signal-to-noise ratio.

Method	PSNR
CNN-15	28.63
Based on *l*_0_ norm	28.32
DEBLURGAN	29.96
SRN	29.57
Algorithm	30.04

**Table 2:** Situation of the case studied.

Occurrence site	Proximal radius	Shoulder blade	Pelvis	Rib cage
Number of cases	4	4	2	2

## Data Availability

The image data used to support the findings of this study are available from the corresponding author upon request.
